The article "Harmine suppresses hyper-activated Ras–MAPK pathway by selectively targeting oncogenic mutated Ras/Raf in Caenorhabditis elegans" was published in 2019. Journal: Cancer Cell Int.

# Harmine suppresses hyper-activated Ras–MAPK pathway by selectively targeting oncogenic mutated Ras/Raf in *Caenorhabditis elegans*

**DOI:** 10.1186/s12935-019-0880-4

**Published:** 2019-06-11

**Authors:** Jiaojiao Ji, Jiang Yuan, Xiaoyu Guo, Ruifang Ji, Qinghua Quan, Mei Ding, Xia Li, Yonggang Liu

**Affiliations:** 1 Beijing University of Chinese Medicine, Beijing, China; 2 State Key Laboratory of Molecular Developmental Biology, Institute of Genetics and Developmental Biology, Chinese Academy of Sciences, Beijing, China

**Keywords:** Harmine, LET-60/Ras, LIN-45/Raf, MAPK pathway, *C. elegans*

## Abstract

**Background:**

Mutationally activated Ras proteins are closely linked to a wide variety of human cancers. Hence, there has been an intensive search for anti-Ras therapies for cancer treatment. The sole Ras gene, which encodes LET-60, in *Caenorhabditis elegans* regulates vulval development. While the loss of *let*-*60* function leads to failure of vulva formation, the *let*-*60*(*n1046gf*) allele, which contains a missense mutation mimicking a Ras codon 13 mutation found in human cancers, results in extra vulval tissue, a phenotype named Muv (multiple vulvas).

**Methods:**

By taking advantage of the easy-to-score Muv phenotype of *let*-*60*(*n1046gf*), we used a step-by-step screening approach (from crude extract to active fraction to active natural compound) to search for inhibitors of oncogenic Ras. Mutants of other key components in the Ras–mitogen-activated protein kinase (MAPK) pathway were used to identify other candidate targets.

**Results:**

The natural compound harmine, isolated from the plant *Peganum harmala*, was found to suppress the Muv phenotype of *let*-*60*(*n1046gf*). In addition, harmine targets the hyper-activation of the Ras/MAPK pathway specifically caused by overexpression or mutated forms of LET-60/Ras and its immediate downstream molecule LIN-45/Raf. Finally, harmine can be absorbed into the worm body and probably functions in its native form, rather than requiring metabolic activation.

**Conclusion:**

In sum, we have revealed for the first time the anti-Ras activity of harmine in a *C. elegans* model system. Our results revealed the potential anti-cancer mechanism of harmine, which may be useful for the treatment of specific human cancers that are associated with oncogenic Ras mutations.

## Background

*Ras* genes were identified initially as retroviral oncogenes. The Ras family consists of four related guanosine triphosphate (GTP)-binding proteins, termed H-Ras, K-Ras, N-Ras, and R-Ras, that play important roles in cell proliferation, differentiation, vesicular trafficking, and gene expression [1, 2]. Wild-type Ras proteins cycle between the GTP-bound (active) and GDP-bound (inactive) states. Ras guanine nucleotide exchange factors (GEFs) promote the formation of Ras-GTP and GTPase-activating proteins (GAPs) that convert GTP-Ras to inactive GDP-Ras [3]. Ras activation is closely linked to 33% of human cancers, making it one of the most frequent oncogenic mutations [4]. Current data reveal that K-Ras is the most frequently mutated Ras in human cancers (21.6%), whereas mutations in H-Ras are the least common (3.3%), followed by mutations in N-Ras (8.0%) [5]. Mutation of codon 12 was first identified as the mechanism underlying K-Ras activation in lung and colon tumor cells [6]. Subsequent studies that combined NIH/3T3 cell transfection assays and DNA sequencing detected activated Ras proteins in a wide spectrum of human tumor cell lines as well as in human patient tumor samples. Ras mutations were later also identified at codons 13 and 61. Although mutations affecting other regions of the proteins have been found, changes at these three codons (12, 13, and 61) account for 97–99% of all Ras mutations in cancer. Among the Ras isoforms, missense mutations are found most commonly in K-Ras (85%), less commonly in N-Ras (12%), and rarely in H-Ras (3%) [2].

Mutations of glutamine 61 (Q61) impair the GTP hydrolysis activity of Ras by interfering with the coordination of the water molecule required for nucleophilic attack on the γ-phosphate of GTP [7, 8]. Oncogenic substitutions at codons glycine 12 (G12) or glycine 13 (G13) prevent the formation of van der Waals bonds between Ras and GAP, thus perturbing the proper orientation of the catalytic glutamine (Q61) in Ras and finally resulting in marked attenuation of GTP hydrolysis [9]. Considering that the mutations identified at different sites in different Ras isoforms all appear to produce constitutively activated Ras proteins, molecules or compounds that inhibit oncogenic Ras activity may serve as anti-cancer therapies for tumors involving Ras mutations [10].

The *let*-*60* gene encodes the sole Ras protein in *Caenorhabditis elegan*s and regulates the formation of the vulva, the egg-laying organ in worms [11]. In wild-type animals, only one vulva develops from the posterior daughter cells of a set of ectodermal P cells (Pn.p cells). There are six vulval precursor cells, P3.p to P8.p. Among them, only P5.p, P6.p, and P7.p can differentiate into vulva tissue, while the other three become hypodermal cells. Loss-of-function (*lf*) mutations in *let*-*60* generate a no-vulva phenotype (Vulvaless or Vul), and gain-of-function (*gf*) mutations in *let*-*60* lead to extra vulval tissue (Multivulva or Muv) [12]. Genetic screens for mutants displaying phenotypes similar to those of various *let*-*60* animals have identified a series of conserved core components in the Ras pathway as well as numerous regulators or targets of the pathway. In fact, many important Ras pathway genes were first identified in worms. Upon growth factor binding, receptor tyrosinase kinases (RTKs) such as LET-23 or EGL-15 form dimers and mutually phosphorylate the C-terminal region of the receptor protein. The phosphorylated tyrosine residues can serve as docking sites for adaptor proteins such as sex muscle abnormal protein 5 (growth factor receptor-bound protein 2) or suppressor of constans overexpression 1 (similar to GRB2-associated binding protein 1). These adaptors subsequently recruit the GEF molecule salt overly sensitive 1 to activate LET-60/Ras. GTP-bound activated LET-60 then binds to LIN-45 Raf and promotes its association with the plasma membrane, endomembranes, or both, on which the LIN-45 kinase can be activated [13]. The scaffold protein kinase suppressor of Ras may assist LIN-45 activation but also promotes further signal transmission by recruiting other mitogen-activated protein kinase (MAPK) cascade components. LIN-45 phosphorylates and activates mitogen-activated protein kinase kinase 2 (MEK-2), MEK-2 then activates mitogen-activated protein kinase 1 (MPK-1), and finally MPK-1 activates or inactivates various target proteins by phosphorylation [14]. MPK-1 can also translocate into the nucleus to phosphorylate transcription factors, such as LIN-1, to alter gene expression (Fig. 1).

**Fig. 1:** The vulval differentiation pathway, mediated by *let*-*60* Ras in *C. elegans*, compared with the Ras-mediated signal transduction pathway controlling mammalian cell division

The *let*-*60*(*n1046gf*) allele encodes a LET-60 protein with the missense mutation G13E (glycine to glutamic acid), which mimics the Ras mutations at codon 13 in many human cancers [12]. In addition to the normal vulva, multiple ectopic vulval-like protrusions are formed along the ventral side of *let*-*60*(*n1046gf*) mutant adults. Here, by taking advantage of the easy-to-score Muv phenotype of *let*-*60*(*n1046gf*), we screened crude extracts from over 30 different species including plants and two animals, and found that the crude extract from *Peganum harmala* effectively inhibits the Muv phenotype of *let*-*60*(*n1046gf*) animals. We further showed that harmine, one of the beta-carboline alkaloids from *P. harmala* (harmal) seeds, could inhibit the activity of the *n1046* mutant form of Ras, but not the wild-type Ras. Among the components of the Ras/MAPK pathway, harmine specifically targets mutated Ras and Raf. Together, our results revealed the potential anti-cancer mechanism of harmine, which may be useful for the treatment of specific human cancers that are associated with Ras mutations.

## Materials and methods

### *C. elegans* genetic stocks

Worms were maintained and manipulated using standard methods as described by Brenner [15]. In brief, worms were cultured on 3-cm nematode growth medium (NGM) plates at 22 °C with OP50 *Escherichia coli* as food unless otherwise mentioned. Mutants and transgenic strains used in this study include the following: LGII, *let*-*23*(*sa62*); LGIV, *let*-*60*(*n1046gf*), *let*-*60*(*n1700gf*), *let*-*60*(*ga89gf*), *lin*-*1*(*e1777*), *kuIs57*(*Pcol*-*10*::LIN-45-AA(S312A/S453A), *Psur*-*5*::GFP); and LGX, *lin*-*15B&lin*-*15A* (*n765ts*). The *kuIs57* mutant was isolated from strain MH2211: *unc*-*29*(*e1072*); *sur*-*6*(*ku123*); kuIs57. All of these strains were obtained from the Caenorhabditis Genetics Center (St. Paul, MN) except for *kuIs12* and *sqt*-*1*;*jgIs25.* The *kuIs12*(*Plet*-*60::let*-*60 wt*) strain was a generous gift from Dr. Min Han (University of Colorado Boulder), and *sqt*-*1*;*jgIs25*(*Plet*-*23*::LET-23::hEGFR-TK [T790M–L858R]), *rol*-*6*(*su1006*) was kindly provided by Dr. Jaegal Shim (National Cancer Center, Goyang, Korea).

### Active compound extraction procedure

To obtain total extracts from 30 species including plants and two animals for screening, 500 ml 70% ethanol (EtOH) was added to 100 g of dried plant and reflux extraction was carried out for 1.5 h using a Soxhlet extractor. The extracts were dried in a flask in a water bath at 95 °C, dissolved in dimethyl sulfoxide (DMSO) to obtain a stock solution of 50 mg total extract per ml, and stored at 4 °C until analysis.

To isolate fractions from *P. harmala* L. seeds, solvents with polarity ranging from low to high, including petroleum ether (PEth), dichloromethane (DCM), ethyl acetate (EtOAc), methanol (MeOH), and water (100 ml each) were added sequentially to 20 g seeds over 4 h for reflux extraction with a Soxhlet extractor. Excess solvent was removed using a rotary evaporator, and the evaporated fractions were then dried in a vacuum desiccator and redissolved in the corresponding isolation solvent (except for the DCM, EtOAc, and MeOH fractions, which were dissolved in DMSO) to obtain a stock solution of 50 mg dried fraction per ml. All of the stocks were stored at 4 °C until analysis.

### Preparation of compounds to test for anti-Ras activity

Harmine, harmol, and harmaline were isolated from the seeds of *P. harmala* L. (provided by Xinjiang Medical University, Urumqi, China) in our lab (School of Chinese Materia Medica, Beijing University of Chinese Medicine, Beijing, China). Dried seeds of *P. harmala* L. (2 kg) were crushed and degreased three times with 3 volumes of PEth for 2 h. The residue was soaked in 5 volumes of cold ammonia water (pH 10–11) for 24 h, and subsequently immersed in 5 volumes of acetic acid solution (pH 3–4) overnight. Residues were removed from the solution by filtering between each treatment. The acetic acid solution was collected, adjusted to pH 12 with ammonia water, and allowed to sit for 24–48 h to obtain a total alkaloid precipitate by filtration.

The total alkaloids (100 g) were dried in a vacuum desiccator and dissolved in MeOH, mixed with 1.2-fold volume of silica gel (200–300 mesh), and subjected to silica gel column chromatography. The total alkaloids were eluted with CH_2_CL_2_:CH_3_OH (20:1), and eluent was collected and the components in the eluent were resolved and detected using silica gel thin-layer chromatography (TLC). Eluents with purple or green fluorescence detected by TLC were combined and allowed to volatilize to dryness. The residue was crystallized in MeTH to obtain a crude compound, which was then subjected to repeated column chromatography and recrystallization to yield harmine and harmaline. Harmol was obtained through the metabolism of harmine by liver microparticles, and was then detected by high-performance liquid chromatography (HPLC)–tandem mass spectrometry (LC–MS–MS). Chemical structures were identified using analytical methods including HPLC, ultraviolet spectroscopy, nuclear magnetic resonance, and MS. The purity of each isolate was > 98% as determined by HPLC. For all worm assays, stock 50 mM solutions of all separated compounds in DMSO and a 10-mM solution of tipifarnib, a farnesyltransferase inhibitor (> 98%; AbMole BioScience, TX) in DMSO were prepared and stored at 4 °C until used for analyses.

### Assays of experimental compounds and phenotypic analysis

To guarantee sufficient exposure to each compound analyzed, both the NGM plates and the OP50 bacteria were supplemented with the experimental compounds (drugs) being tested. Either vehicle (DMSO solvent) alone or vehicle plus experimental drug (*P. harmala* extracts, tipifarnib, harmine, harmaline, or harmol) was mixed with the NGM just before pouring into 3-cm diameter plates to achieve the final desired concentration (dose). Plates were held at room temperature until the agar solidified, and then were kept at 4 °C for up to 7 days. On day 0, approximately 80–100 gravid worms were chosen and allowed to lay eggs for 2 h to obtain synchronized embryos, after which the parents were removed from the plate. A 20-μl mixture of drug or vehicle along with concentrated dead OP50 suspended in M9 buffer was immediately added to the synchronized embryos on each plate. To prepare dead OP50 to avoid metabolism of the drugs by bacteria, 200 ml OP50 bacteria suspension in LB media was centrifuged at 8000 rpm for 10 min. The bacterial pellet was then resuspended in 20 ml M9 buffer and killed at 65 °C for 2 h. After hatching, the worms were cultured for 3–4 days at 22 °C. Day 1 adults bearing 2–8 eggs were mounted on slides in M9 buffer containing 1% 1-phenoxy-2-propanol to score the percentage of Muv animals and number of ectopic vulvas per animal using a Zeiss imager A1 upright microscope at 20× magnification. The criteria for recognition of the Muv phenotype have been described by Horvitz and Sulston. Adults with one or more pseudovulvas (ventral protrusions) in addition to a normal vulva were classified as Muv. The assay for each test compound was repeated at least three times; over 100 worms per experiment and dose were observed to statistically analyze Muv phenotype.

In the experiments with the temperature-sensitive *let*-*60*(*ga89*) mutant, which has a germ-line developmental defect such that small immature oocytes stack irregularly in the proximal gonad arm, synchronized embryos were grown at 16 °C for 90 h until larval stage 4 (L4 stage). The percentage of animals with abnormal gonads was calculated after worms were shifted to 25 °C for 12 h.

### Ultra-performance liquid chromatography-multi-stage MS analyses and sample preparation

Worms treated with 160 μM harmine- or 0.8% DMSO-were collected and washed three times with aseptic M9 solution in 15 ml Corning tubes. The worm pellet was completely homogenized using a Dounce homogenizer (Cheng-He, Zhuhai, China) in a 75% MeOH–water solution and processed by ultrasonication for 10 min after the homogenates were transferred to 1.5 ml microfuge tubes. The supernatant was injected into vials after centrifugation at 13,000 rpm for 15 min. Finally, 2 μl of sample from each group was injected into an ultra-performance liquid chromatography quadrupole time-of-flight multi-stage MS (UPLC-Q-TOF-MS^n^) apparatus for analysis. Separation and analysis of the samples were performed on a Waters ACQUITY™ UPLC I-Class system (Waters, USA) equipped with a binary solvent system. The system was controlled using MassLynx V4.1 software. Sample separation was achieved on an ACQUITY BEH C_18_ column (1.7 μm, 2.1 × 100 mm; Waters, UK) at 40 °C with a flow rate of 0.4 ml/min. For separation of DCM or EtOAc extracts from *P. harmala*, the mobile phase was composed of 0.1% (v/v) formic acid in water (A) and acetonitrile (B) with a gradient program: 0–6 min, 1–50% B; 6–12 min, 50–60% B; 12–13 min, 60–85% B; 13–14 min, 85% B. For separation of worm extracts, the mobile phase was composed of 0.1% (v/v) formic acid in water (A) and acetonitrile (B) with a gradient program: ~ 0–13 min, 1–95% B; 13–14 min, 95% B.

MS data were recorded using the Waters SYNAPT G2-SI MS^E^ system (Waters) equipped with an electrospray ionization source and Q-TOF-MS/MS. The three-dimensional data were collected in the continuum mode. The optimized source parameters in positive ion mode were set as follows: capillary voltage, 3.0 kV; sampling cone voltage, 40 V; source offset, 50; source temperature, 100 °C; desolvation temperature, 400 °C; desolvation gas flows, 800 l/h; nebulizer, 7.0 bar. Collision energy of the low energy function was set at 6 V, and the ramp trap collision energy of the high energy function was set at 10–40 V. Data were collected from *m/z* 100 to 1200 Da. Leucine-enkephalin (*m/z* 556.2771 in positive ion mode) was used as the external mass reference and was infused using a LockSpray™ source at a constant flow rate of 5 μl/min. The mass spectrometer was calibrated over a range of 100–1200 Da with sodium formate. Data analysis was performed using MassLynx V4.1 software and UNIFI™ 1.7 software from Waters (based on an in-house traditional Chinese medicine database).

### Western blots

Gravid worms were transferred to new NGM plates to lay eggs for 2 h, then 800–1000 eggs were transferred to duplicate 6-cm NGM plates supplemented with 0.8% DMSO as control or other compounds including tipifarnib (160 μM), harmine (160 μM), harmaline (320 μM), or harmol (320 μM) in both the medium and heat-killed OP50 *E. coli*. Hatched worms were cultured in an incubator at 22 °C until the L4 stage. Worms were collected and washed twice with M9 buffer in 15-ml Corning tubes (Corning Costar, Corning, NY) to remove bacteria and worms were allowed to settle in the tubes naturally. Supernatants were removed, about 1 ml of worm suspension was pipetted into 1.5-ml microfuge tubes, and the tubes were centrifuged at 8000 rpm for 2 min to pellet worms. The supernatants were then removed. Then, 50–90 μl of lysis buffer (50 mM Tris–HCl pH 7.5, 150 mM NaCl, 1 mM EDTA, 0.2 mM dithiothreitol [DTT], 1% Triton X-100, v/v; 10% glycerol, v/v) supplemented with protease inhibitor (#04693132001, Roche, Mannheim, Germany) and 1 mM phenylmethylsulfonyl fluoride was added to the worm pellet. After grinding for 5 min on ice with a motorized tissue grinder (#G50, Ginkgo), worm lysates were centrifuged at 13,000 rpm for 10 min at 4 °C. Supernatants were transferred to new 1.5-ml microfuge tubes and protein concentrations was detected using a Pierce BCA Protein Assay Kit (#23225, Thermo Fisher Scientific, Waltham, MA). Equal amounts of total proteins (35 μg) were subjected to electrophoresis after being boiled at 100 °C with 5× sodium dodecyl sulfate sample buffer containing 100 μM DTT. The proteins were then transferred to nitrocellulose membranes. The membranes were then blocked in 5% non-fat milk at room temperature for 1 h and were then incubated with anti-Ras (#EPR3255, Abcam, Cambridge, MA) or anti-α-tubulin (#T6074, Sigma-Aldrich, St. Louis, MO) first antibody at 4 °C overnight. Next, membranes were incubated with goat anti-rabbit/anti-mouse secondary antibody conjugated with horseradish peroxidase (1:5000) in 5% non-fat milk for 1 h. Membranes were washed three times before and after second antibody incubation with 1× Tris-buffered saline with Tween 20 for 15 min each time. After Pierce ECL Western Blotting Substrate (#32106, Thermo Fisher Scientific) was added to the membranes, the protein bands were visualized using a mini chemiluminescence imaging system (MiniChemi™ 500, Saizhi, Beijing, China).

### Statistical analysis

In this study, data were derived from at least three independent experiments in which over 300 worms were counted at day 1 adult stage when scoring the Muv phenotype. Data were analyzed using a Student’s t-test or one-way analysis of variance to compare differences in values between the control and experimental groups. The results are presented as the mean ± standard deviation, where *p* < 0.05 indicated a statistically significant difference.

## Results

### Tipifarnib suppresses both the *n1046* mutant and wild-type LET-60/Ras

To test whether *let*-*60*(*n1046*) can serve as a drug screen model system in *C. elegans*, we investigated the ability of a known anti-Ras reagent to suppress the Muv phenotype. Ras proteins require lipid modification to be inserted into the plasma membrane where they perform their functions (Fig. 1) [16]. Interestingly, previous studies found that the Ras farnesyltransferase inhibitors manumycin and gliotoxin efficiently inhibited the Muv phenotype of *let*-*60*(*n1046*) [10]. This supports the notion that the mutant *let*-*60*(*n1046*) indeed encodes a hyper-active or constitutively activated Ras protein, and that the Muv phenotype of *let*-*60*(*n1046*) can serve as a drug screening model system. Tipifarnib (also named R115777, Fig. 2a) is an imidazole farnesyltransferase inhibitor that is in Phase III clinical trials [5]. When we treated *let*-*60*(*n1046*) animals with 0.8% DMSO (control) or different doses of tipifarnib, the number of Muv animals in the *let*-*60*(*n1046*) population dose-dependently decreased when treated with tipifarnib compared with DMSO (80.9%, n = 286) (Fig. 2b, c). Overexpression of a wild-type copy of the *let*-*60* gene also led to a Muv phenotype (75.5%, n = 319) (Fig. 2d, upper panel, and e). When *let*-*60* overexpression animals (*kuIs12*) were treated with 80 μM tipifarnib, the Muv phenotype was also significantly suppressed (23.3%, n = 331) (Fig. 2d lower panel, and e). Thus, Muv animals resulting from either a *gf* mutation in *let*-*60*(*n1046*) or overexpression of the *let*-*60* gene can serve as a valuable system with which to screen for compounds with Ras pathway inhibition activity.

**Fig. 2:** The Muv phenotype caused by LET-60 Ras overactivation is suppressed by the farnesylation inhibitor tipifarnib. **a** Structure of tipifarnib. **b** The Muv phenotype in *let*-*60*(*n1046gf*) is suppressed dose-dependently by tipifarnib treatment. **d** In *kuIs12*, 80 μM tipifarnib could suppress the Muv phenotype significantly as well. Statistical analysis of the Muv ratio and the number of ectopic vulvas are shown in **c** and **e**, respectively. White arrows indicate pseudovulvas and black arrowheads indicate normal vulvas. *p < 0.05; **p < 0.01; ***p < 0.001 by unpaired Student’s *t*-test

### Identification of potential Ras pathway inhibitors from plant extracts

Next, we screened plant extracts to identify putative Ras pathway inhibitors using the Muv *let*-*60*(*n1046gf*) mutant animals as a model system. EtOH extract (5 mg/ml, 70%) from individual plants was mixed with heat-killed OP50 bacteria and the mixture was placed on NGM plates to feed *let*-*60*(*n1046*) animals. From extracts of about 30 species tested (Table 1), we found that the extract from seeds of *P. harmala* significantly suppressed the Muv phenotype of *let*-*60*(*n1046*). Even when the extract concentration was decreased to 500 μg/ml, the 70% EtOH extract from *P. harmala* seeds still efficiently inhibited the Muv phenotype of *let*-*60*(*n1046*) (from 97.7%, n = 305, to 14.2%, n = 315) (Fig. 3a). In addition, the average number of ectopic vulvas per animal decreased from 2.0 to 0.2 when treated with the *P. harmala* extract. Next, different fractions were extracted from *P. harmala* seeds using solvents ranging from low to high polarity, including PEth, DCM, EtOAc, MeOH, and water. When *let*-*60*(*n1046*) animals were fed dead OP50 treated with these fractions (500 μg/ml), we found that the DCM and EtOAc extracts specifically suppressed the Muv phenotype of *let*-*60*(*n1046*) (Fig. 3b).

**Table 1:** Thirty medicines used to screen for anti-Ras activity in *C. elegans*

	Medicines
1	Radix Astragali
2	Semen Cuscutae
3	*Peganum harmala*
4	*Portulaca oleracea*
5	Radix Angelicae Sinensis
6	Fructus Aurantii Immaturus
7	Radix Aconiti Kusnezoffii
8	Rhizoma Coptidis
9	*Crataegus pinnatifida*
10	Monkshood
11	*Tribulus Terrestris*
12	*Piper kadsura*
13	*Codonopsis pilosula*
14	*Lycium chinense*
15	Radix Aucklandiae
16	Tangerine Peel
17	Rhizoma Zingiberis
18	*Asparagus*
19	Great Burdock
20	Common *Bletilla* Tuber
21	*Pheretima aspergillum* (E. Perrier)
22	Folia Bambosae
23	Scorpio
24	*Platycladus orientalis*
25	Herba Lycopi
26	*Rhynchophylla*
27	Semen Nelumbinis
28	*Codonopsis pilosula*
29	Rhizoma Polygonati
30	*Ginkgo biloba*

**Fig. 3:** Screening of extracts of plant and animals reveals that the DCM and EtOAc fractions of *P. harmala* seed extracts inhibit the Muv phenotype in *let*-*60*(*n1046gf*). **a** 70% EtOH extract of *P. harmala* seeds suppresses the Muv phenotype in *let*-*60*(*n1046gf*). White arrows indicate pseudovulvas and black arrowheads indicate normal vulvas. Statistical analyses of the data are also shown. **b** TLC results showed that the 70% EtOH extract contained harmine. **c** Among five fractions, the DCM and EtOAc fractions of *P. harmala* significantly inhibit the Muv phenotype. **d** TLC of five fractions from *P. harmala* seeds and harmine standard. ***p < 0.001 by unpaired Student’s *t*-test

To identify potential active components in the *P. harmala* extract, silicon TLC was used to analyze the DCM and EtOAc fractions. Interestingly, we found that harmine, one of the most abundant alkaloids in *P. harmala* seeds [17], was present in the 70% EtOH total extract (Fig. 3c) as well as the DCM and EtOAc fractions, but little or none was present in the other three fractions (Fig. 3d). Using the UPLC-MS^n^ technique, we further analyzed the compounds in the DCM and EtOAc extracts. Consistent with the TLC data, the same peak corresponding to the most abundant component appeared in both fractions in the base peak ion chromatograph (positive ion mode). Based upon the characterized MS fragments (*m/z* 213.1016, 198.0790, 170.0850, 144.0811), this peak very likely corresponds to harmine (Fig. 4a, b). In addition to harmine, peaks corresponding to vasicine, desoxypeganine, and vasicinone were recognizable in both the DCM and EtOAc fractions, but the relative abundance of these three compounds was low.

**Fig. 4:** Harmine is the most abundant compound in both DCM and EtOAc fractions. **a** and **b** Base peak ion chromatogram (BPI) analysis of the DCM and EtOAc fraction in positive ion mode. The highest peak was analyzed and the MS spectrum in a higher energy scan is shown in the upper rectangle. Both fractions share similar BPI patterns, and the most abundant component is harmine

### Harmine treatment suppresses the Muv phenotype of *let*-*60*(*n1046gf*)

Harmine belongs to the β-carboline alkaloid family of compounds and is highly enriched in *P. harmala* seeds. Harmine has been shown to possess anti-cancer potential in various cancer cell lines [18–21] and in mice models with explanted tumor tissues [22]. However, it has not previously been shown whether harmine functions as a Ras inhibitor to suppress tumor growth. Two harmine-related β-carboline alkaloids, harmaline and harmol, were also isolated from *P harmala* seeds (Fig. 5a). We next tested the three β-carboline alkaloids to determine which one showed Muv inhibition activity. Intriguingly, while harmine treatment significantly decreased the Muv phenotype of *let*-*60*(*n1046*) mutant worms, neither harmaline nor harmol showed such suppression of the *let*-*60*(*n1046*) phenotype (Fig. 5b).

**Fig. 5:** Harmine is the active Muv-suppressive component in the DCM and EtOAc fractions. **a** Structures of harmine, harmaline, and harmol. **b** Only harmine treatment suppresses the Muv phenotype in *let*-*60*(*n1046gf*). **c** Harmine reduces the percentage of Muv animals and the number of ectopic vulvas is in a dose-dependent manner. **d** and **e** Harmaline and harmol have little effect on the Muv phenotype in *let*-*60*(*n1046gf*). White arrows indicate pseudovulvas and black arrowheads indicate normal vulvas. *p < 0.05; **p < 0.01; ***p < 0.001 by one-way analysis of variance

We next tested whether harmine inhibits the *let*-*60*(*n1046gf*) Muv phenotype in a dose-dependent manner. We treated *let*-*60*(*n1046gf*) animals with different concentrations of harmine and found that the Muv suppression efficiency of harmine increased at higher concentrations (Fig. 5c), whereas increasing doses of harmaline and harmol showed little or no suppressive effect (Fig. 5d, e). We further examined whether suppression of the Muv phenotype by harmine could be transduced to the next generation. When harmine-treated non-Muv *let*-*60*(*n1046gf*) animals (n = 5, one worm/plate) were transferred to NGM plates containing no harmine and allowed to lay eggs, we found that most of the newly hatched animals exhibited the Muv phenotype upon reaching adulthood, similar to control animals that had not been treated with harmine (~ 80%) (data not shown). Thus, the Muv inhibition activity of harmine is not heritable.

### Harmine likely functions to inhibit the Muv phenotype of *let*-*60*(*n1046*) in its native form

To address whether harmine inhibits Muv of *let*-*60*(*n1046*) in its native form or through its metabolites when consumed by worms, we used UPLC-Q-TOF-MS to analyze the compounds and metabolites present in harmine- and mock (DMSO)-treated *let*-*60*(*n1046*) animals. A characteristic peak (*m/z* 213.1016) (Fig. 6b, lower panel) with MS fragments of *m/z* 198.0790, 170.0850, and 144.0811 (Fig. 6b, upper rectangle) appears specifically in harmine-treated worms. We noticed that these MS fragments are consistent with the fragments typical of harmine in positive ion mode. In contrast, when we searched for characteristic peaks indicating the existence of harmine metabolites, for instance harmol, we found no such peaks in the harmine-treated animals. Together, these results suggest that harmine likely functions in its native form in worms to inhibit the Muv phenotype of *let*-*60*(*n1046gf*).

**Fig. 6:** Harmine functions in its native form to suppress the Muv phenotype. BPI of extracts of worms treated with either 0.4% DMSO vehicle (**a**) or 80 μM harmine (lower panel, **b**). The chromatogram contains a new peak, *m*/*z* 213 (indicated by a red line). The MS spectrum of a higher energy scan is shown (upper rectangle, **b**) and indicates the existence of harmine, but not metabolites of harmine, inside the worm body

### Harmine does not suppress the Muv phenotype caused by overexpression of wild-type LET-60

The *let*-*60*(*n1046gf*) mutation causes a missense mutation at codon 13 (G13E) that is analogous to the frequently observed mutation in the human K-Ras protein in malignancies. To rule out the possibility that harmine-induced suppression of the Muv phenotype is due to the genetic background in *n1046*, we tested harmine function in another *let*-*60* allele, *n1700*, which contains the same G13E mutation as n1046 [11]. Similar to *n1046*, the Muv phenotype is highly penetrant in *n1700*. When treated with the compounds and drugs described above, the Muv ratio in *n1700* was suppressed strongly by harmine and moderately by tipifarnib, while harmaline and harmol treatment had almost no effect (Fig. 7a, b), which is consistent with the previous data from *n1046*, implying that harmine is more likely to target LET-60/Ras overactivation caused by the G13E mutation but not by the genetic background.

**Fig. 7:** Harmine reverses the phenotype induced by a LET-60 hyper-activating mutation. **a** and **b** Harmine treatment could suppress the Muv phenotype in *let*-*60*(*n1700gf*). **c** and **d** Harmine suppresses the abnormal gonad phenotype (small stacked oocytes) in the LET-60 hyper-activation mutation strain *let*-*60*(*ga89gf*). Red lines in **c** outline the oocytes. White arrows indicate pseudovulvas and black arrowheads indicate normal vulvas. **p < 0.01; ***p < 0.001 by unpaired Student’s *t*-test

In order to test whether the Muv-suppressive effect of harmine is allele-specific, we tested *let*-*60*(*ga89*) mutant animals. The *ga89* mutant has a leucine (L) to phenylalanine (F) mutation at amino acid 19 in LET-60 [23]. It was reported that this mutation results in a temperature-sensitive phenotype in worms: at the lower temperature of 15 °C, the Ras activity of LET-60 remains relatively normal and the animals display no obvious morphological defects, whereas at 25 °C, LET-60 activity increases and about 38% of animals display a weak Muv phenotype. In addition, small irregular immature oocytes become stacked in the proximal gonad arm of *let*-*60*(*ga89*) animals at 25 °C [24] (Fig. 7c, upper panel). However, when the animals were treated with 80 μM harmine, the oocyte underdevelopment phenotype of *let*-*60*(*ga89*) was significantly suppressed, and tipifarnib also showed some suppressive activity, while harmaline and harmol had no effect (Fig. 7c, d). The above data suggest that harmine can inhibit the abnormal Ras activity caused by the *let*-*60*(*ga89*) mutation.

After showing that harmine can suppress the Muv phenotype induced by the codon 13 mutation in *let*-*60*(*n1046gf*) and oocyte underdevelopment phenotype caused by the codon 19 mutation in the Ras-like LET-60 encoded by of *let*-*60*(*ga89*), we wondered whether harmine specifically affect mutationally activated Ras or whether it inhibits Ras activity in general. Previous studies have shown that overexpression of the wild-type *let*-*60* gene also induces extra vulval tissue [25]. Therefore, we tested the inhibitory effect of harmine on the Muv phenotype induced by *let*-*60*-overexpression. Interestingly, similar to harmaline and harmol, treatment with harmine, even at a high concentration (160 μM), did not suppress the Muv phenotype in the *let*-*60* overexpression animals (Fig. 8a, b). Unlike the farnesyltransferase inhibitor tipifarnib, which suppressed the Muv phenotype induced by both the *let*-*60*(*n1046gf*) mutation and *let*-*60* overexpression, harmine seems to exhibit some selectivity in terms of targeting the mutated form of Ras proteins rather than the wild-type form.

**Fig. 8:** Harmine treatment could not suppress the Muv phenotype in wild-type *let*-*60* overexpression animals. **a** and **b** Harmine treatment has no effect on the Muv phenotype of *kuIs12*, a wild-type *let*-*60* overexpression strain. White arrows indicate pseudovulvas and black arrowheads indicate normal vulvas. **p < 0.01; ***p < 0.001 by unpaired Student’s *t*-test

### Harmine selectively targets components of the Ras/MAPK signaling pathway

We next asked whether harmine could affect other components of the Ras/MAPK signaling pathway. LIN-45/Raf is the direct downstream binding partner of LET-60/Ras (Fig. 1), and is recruited to the cell membrane by Ras through its Ras-binding domain [26]. Overexpression of mutant LIN-45/Raf-AA (S312A/S453A) causes excessive activated Ras/MAPK signaling and leads to the Muv phenotype in worms [25]. When the LIN-45/Raf-AA (S312A/S453A) overexpression animals were treated with harmine, we found that the Muv phenotype was significantly suppressed (from 82.3 to 24.8%) (Fig. 9a, b).

**Fig. 9:** Harmine could suppress Muv phenotype on some components of the LET-60 signaling pathway. **a** and **b** Harmine inhibits the Muv phenotype in *kuIs57*, a strain that overexpresses the *lin*-*45* hyperactivation mutation LIN-45-AA (S312A/S453A). **c** and **d** Harmine has no effect on *let*-*23*(*sa62*) mutants, with a *gf* mutation in EGFR. **e** and **f** Harmine moderately decreases the percentage of Muv animals and the number of ectopic vulvas in *jgIs25*, a transgenic strain overexpressing a chimeric protein consisting of the LET-23 N-terminus and the human EGFR C-terminus carrying the tyrosine kinase mutations T790M–L858R. White arrows indicate pseudovulvas and black arrowheads indicate normal vulvas. *p < 0.05; **p < 0.01; ***p < 0.001 by unpaired Student’s *t*-test

The *let*-*23* gene encodes the epidermal growth factor receptor (EGFR) in *C. elegans*, which functions upstream of LET-60/Ras. Along the same lines, the *gf let*-*23*(*sa62*) mutation also results in a Muv phenotype. Interestingly, harmine treatment did not suppress the Muv phenotype of *let*-*23*(*sa62*) (Fig. 9c, d). Further, we examined the effect of harmine on the Muv phenotype in *jgIs25* animals, which express a chimeric protein created by fusing the N-terminus of LET-23 with the C-terminus of human EGFR. The EGFR portion contains two missense mutations (T790M–L858R) in the tyrosine kinase domain that have been identified in human cancers. The expression of this chimeric protein in *C. elegans* vulva tissue also leads to a Muv phenotype [27]. We found that when *jgIs25* worms were fed with harmine, the Muv phenotype was marginally suppressed (Fig. 9e, f).

LIN-15 acts on hypodermal cells and negatively regulates the Ras/MAPK signaling pathway. The *lin*-*15*(*n765ts*) *lf* allele is temperature-sensitive. Thus, 100% of *lin*-*15*(*n765ts*) animals exhibit a Muv phenotype at 22 °C, while 0% display the mutant phenotype at 16 °C [28]. Upon harmine treatment (160 μM), no obvious change was observed in the percentage of Muv animals. However, the average number of ectopic vulvas appeared to be moderately lower with harmine treatment (Fig. 10a, b).

**Fig. 10:** Harmine had little effect on other LET-60 signaling pathway components. **a** and **b** Mild suppression of the number of ectopic vulvas, but not the Muv phenotype, in *lin*-*15*(*n765 ts*) mutants by harmine. **c** and **d** Harmine has no effect on *lin*-*1*(*e1777lf*) mutants. White arrows indicate pseudovulvas and black arrowheads indicate normal vulvas **p < 0.01. **e** Representative western blots of Ras levels in *let*-*60*(*n1046*) treated with tipifarnib (160 μM), harmine (160 μM), harmol (320 μM), or harmaline (320 μM). Harmine treatment had no effect on LET-60/Ras protein level

The *lin*-*1* gene encodes the *C. elegans* homolog of the ETS-domain transcription factor, which is negatively regulated by the Ras/MAPK pathway [29]. The *lin*-*1*(*e1777*) *lf* allele also displays a Muv phenotype. When *lin*-*1*(*e1777*) mutants were fed with harmine (160 μM), no suppression of the Muv phenotype was observed (Fig. 10c, d).

To test whether Muv suppression is due to alteration of the LET-60/Ras protein level, western blot assays were conducted on proteins isolated from the L4 stage (the key stage for vulval development) *let*-*60*(*n1046*) worms treated with different compounds or drugs. Both tipifarnib and harmine, which could suppress the Muv phenotype, had little effect on LET-60/Ras protein abundance (Fig. 10e), indicating that harmine is more likely to function through Ras activity than through regulation of LET-60/Ras protein abundance.

In summary, harmine specifically suppresses the Muv phenotypes caused by *let*-*60*(*n1046gf*) and LIN-45/Raf-AA (S312A/S453A), and suppresses germ-line developmental defects in *let*-*60*(*ga89*), suggesting that harmine only targets some mutationally activated Ras and Raf proteins and may therefore serve as an anti-cancer drug for a specific set of tumors.

## Discussion

Previous studies have suggested that harmine induces cell cycle arrest or apoptosis through (i) intercalation into DNA and inhibition of protein synthesis [30], (ii) inhibition of DNA repair via homologous recombination [21], (iii) down-regulation of the cyclooxygenase-2 protein abundance in gastric cancer [31], (iv) inhibition of the Akt and ERK signaling pathways [19], or (v) inhibition of dual-specificity tyrosine-phosphorylation-regulated kinase 1A [32, 33]. Harmine was also reported to activate p53 and inhibit tumor angiogenesis [34]. In addition, harmine has been reported to inhibit BCRP (breast cancer resistance protein) and reverse resistance to cancer drugs [35]. However, the role of harmine in Ras and Raf inhibition has not previously been revealed.

### *let*-*60*(*n1046gf*) serves as a valuable in vivo drug screening model system

Since first introduced into biological studies as a model organism by Sydney Brenner in the 1960s, *C. elegans* has played a pivotal role in elucidating the functions of genes and genetic pathways that control various important cellular processes. Comparative proteomic studies have revealed that at least 83% of the *C. elegans* proteome has human homologs [36, 37], and 782 out of 2259 human disease genes could be identified in *C. elegans* [38]. Therefore, *C. elegans* has been extensively used to dissect the mechanisms underlying human genetic diseases. More recently, worms have also served as a valuable tool for drug discovery [39–42]. In particular, the worm model has been used to screen for specific inhibitors of double-mutant EGFR [T790M–L858R], which is resistant to the EGFR tyrosine kinase inhibitors gefinitib and erlotinib used in anticancer treatment. The aforementioned study suggested that *C. elegans* could be a useful model system for discovery of EGFR-Ras-MAPK pathway inhibitors. In the present work, *let*-*60*(*n1046gf*) worms were used for the first time as a model system to identify anti-Ras agents. The identification of harmine as a compound that selectively inhibits some mutant hyper-activated Ras and Raf proteins highlights the effectiveness of combining modern analytical chemistry techniques with powerful genetic analysis in *C. elegans*.

Several features of the design of this study are noteworthy. Firstly, the *n1046* mutation (G13E) faithfully mimics the corresponding human mutation, which makes the screen practically meaningful. Second, the distinct Muv phenotype makes the screen relatively easy. Third, the fact that the crude *P. harmala* extract showed significant Muv inhibition implies that drug screening can be performed efficiently in worms using mixtures of many different compounds. Fourth, the huge collection of worm mutants and transgenic lines will be valuable for identifying drugs relevant to humans, given the high conservation between worms and humans in terms of various signaling pathways. Using the CRISPR/Cas9 system oncogenic *Ras* genes could be introduced into *C. elegans* to mimic human disease-causing mutations. In the future, with improvements in high-throughput workflow, imaging platforms, and data analysis software, other drug screens using the Muv-based system in *let*-*60* mutants will become high-efficiency tools to identify more Ras mutation-specific inhibitors.

### Targeting “undruggable” Ras

Ras mutations exist in a variety of cancer types and play an important role in tumor development [43], and even in tumor maintenance [44]. Ras is a molecular switch, and its function relies on its transition between the GTP-binding form (active) and the GDP-binding form (inactive). Oncogenic Ras mutations (at codons 12, 13, and 61) impair GTP-Ras hydrolysis and produce constitutively activated Ras in the absence of extracellular stimuli. The difficulty of developing inhibitors that target Ras directly lies in the picomolar binding affinity of Ras for both GTP and GDP. Thus, Ras has been considered as an “undruggable” protein, and no direct Ras inhibitor has been tested in clinic trials so far. Recently, drugs have been designed based on the specific structure of Ras mutants. These include small molecules that target the mutated cysteine in K-Ras^G12C^ [45], and compound 3144, which targets K-Ras^G12D^ [46]. In our work, harmine exhibits unique selectivity in suppressing the Muv phenotype induced by the *let*-*60*/Ras mutation but not by overexpression of wild-type *let*-*60*. In contrast, tipifarnib, a farnesyltransferase inhibitor, targets both mutated and wild-type Ras. To understand the molecular mechanism of the targeting selectivity of harmine, our future work should include determining the binding affinity between harmine and various Ras mutants as well as wild-type Ras. Computer-aided molecular simulation and crystal structure analysis should also provide valuable information to identify specific oncogenic Ras targeting sites. Of course, harmine could also be structurally modified.

The Raf serine/threonine kinases are key signal transducers in the Ras/MAPK signaling pathway. As a direct effector of Ras, Raf is recruited to the plasma membrane by GTP-bound Ras (active) through direct interactions in which Raf kinase activity is regulated by other factors [47]. There are three Raf members in humans, A-, B-, and C-Raf, among which B-Raf is mutated in approximately 8% of all cancers [48], whereas mutation of the other two Rafs is rare. *BRAF* somatic missense mutations occur in 66% of melanomas, and the most frequent mutation (B-Raf^V600E^) is found in approximately 50% of melanomas, rendering B-Raf inhibitor development an important anticancer strategy. However, one major challenge is to develop more potent inhibitors, such as PLX7904 and PLX8394, which do not evoke paradoxical ERK activation, the unexpected activation of the MAPK pathway after Raf inhibitor treatment [49]. In our study, harmine suppressed the Muv phenotype induced by overexpression of LIN-45gf-AA (S312A/S453A), suggesting that it also has potential as an inhibitor of oncogenic Raf. In the presence of oncogenic Ras, the B-Raf inhibitor PLX4720 and 885-A promotes Ras-dependent B-Raf binding to C-Raf, and activates MEK-ERK signaling [50] to stimulate tumorigenesis. As an inhibitor of both oncogenic Ras and Raf, harmine might overcome the serious side-effects of previous B-Raf inhibitors in patients with both Ras and B-Raf mutations. How does harmine selectively target specific mutated Ras and Raf? Harmine might bind individually to mutated proteins and attenuate their hyper-activation, or disrupt Ras/Raf interactions to restrain signal transduction, which will be tested in our future study.

In addition, harmine could suppress Muv phenotype in the LET-23 hEGFR-TK [T790M–L858R] overexpressing strain, though not strongly, but not in *let*-*23*(*sa62*) animals. The *sa62* gene contains a cysteine 359 to tyrosine mutation in LET-23 EGFR extracellular cysteine-rich domain I, which causes ligand-independent activation of LET-23 EGFR, while hEGFR-TK [T790M–L858R] mutations are located in the intracellular tyrosine kinase domain. The selectivity of harmine might result from differences in the structure and manner of activation of mutated LET-23 EGFR, and could also imply that harmine can function only inside of cells. Further studies are needed to test protein-compound interactions and analyze structural differences in mutated LET-23 to answer this question.

## Conclusion

In summary, harmine acts through Ras-MAPK signaling to regulate vulval formation in *C. elegans*. Moreover, it may selectively suppress mutated Ras/Raf activity, which potentialize it to drug development to treat certain Ras-related cancers in the future.

## Data Availability

All data generated or analyzed during this research are included in this manuscript.

## Abbreviations

DCM: dichloromethane
DMSO: dimethyl sulfoxide
DTT: dithiothreitol
EGFR: epidermal growth factor receptor
EtOAc: ethyl acetate
EtOH: ethanol
G12: glycine 12
G13: glycine 13
GAP: GTPase-activating protein
GEF: guanine nucleotide exchange factor
*gf*: gain of function
GTP: guanosine triphosphate
L4 stage: larval stage 4
*lf*: loss of function
MAPK: mitogen-activated protein kinase
MEK-2: mitogen-activated protein kinase kinase 2
MeOH: methanol
MPK-2: mitogen-activated protein kinase 1
MS/MS: tandem mass spectrometry
Muv: multiple vulvas
NGM: nematode growth media
NSFC: Natural Science Foundation of China
PEth: petroleum ether
RTK: receptor tyrosinase kinase
TLC: thin-layer chromatography
UPLC-Q-TOF-MS^n^: ultra-performance liquid chromatography quadrupole time-of-flight multi-stage mass spectrometry
